# Application of Traditional Chinese Medical Science Characteristic Nursing Mode Based on Evidence-Based Medicine to Puerperal Breast Tenderness and Pain

**DOI:** 10.1155/2022/7527890

**Published:** 2022-06-30

**Authors:** Jingying Liu, Hua Chen, Wei Wang, Dan Zhao

**Affiliations:** ^1^Department of Traditional Chinese Medicine, Taizhou First People's Hospital, Taizhou 318020, Zhejiang, China; ^2^Department of Obstetrics and Gynecology, Taizhou First People's Hospital, Taizhou 318020, Zhejiang, China

## Abstract

**Objective:**

To explore the effects of traditional Chinese medicine (TCM) characteristic nursing mode based on evidence-based medicine on parturients with breast tenderness and pain.

**Method:**

100 parturients with postpartum breast pain treated at Taizhou First People's Hospital from January 2020 to December 2021 were selected. Among them, 51 cases received routine nursing intervention (general group, GG) and 49 cases received TCM characteristic nursing based on evidence-based medicine (comprehensive group, CG). The pain number (NRS) score, lactation effect, breastfeeding self-efficacy (BSES-SF) score, anxiety and depression, and nursing satisfaction of the two groups were compared. In addition, the pregnant women were followed up after discharge to investigate the rate of exclusive breastfeeding.

**Result:**

Three days after intervention, NRS score, SAS score, and SDS score in the CG were significantly lower than those in the GG. The level of serum prolactin and total breast lactation yield in the GG were better than those in the CG. BSES-SF score, nursing satisfaction, and exclusive breastfeeding rate in the CG were higher than those in the GG.

**Conclusion:**

Evidence-based TCM care can significantly reduce postpartum breast tenderness, increase milk production, improve exclusive breastfeeding, and help relieve emotional distress.

## 1. Introduction

Breast tenderness is a common problem in obstetrics, which is caused by the obstruction of milk discharge and the accumulation of milk in the milk ducts after childbirth [1]. If breast distension is not treated in time, it may develop into breast abscess, mastitis, or even systemic infection, which may adversely affect the quality of breast milk and maternal health [2, 3]. At present, most hospitals use traditional massage techniques to unblock the blocked ducts, to promote the discharge of milk, and thus reduce maternal breast distension and pain. However, in actual operation, the phenomenon of “pass again block, block to pass” often occurs, which invariably causes great mental stress and negative emotions to the mothers.

Clinical measures such as postpartum rehabilitation biostimulation feedback instrument, postpartum rehabilitation therapy instrument, and hot compress are used to treat maternal postpartum breast swelling and pain to relieve maternal breast swelling and pain sensation, but the above methods require prolonged intervention and do not have absolute efficiency. With the widespread use of Chinese medicine meridian theory in obstetric rehabilitation care, acupressure through Shaozhe, Quchi, Hegu, Yunmen, and Zhongfu acupoints [4] can, to a certain extent, relieve postpartum breast distension and pain, unblock local blood circulation in the breast, and promote lactation. Cupping therapy is a common treatment method in TCM, and according to the actual situation of mothers after delivery, the main cause of breast distension and pain is stagnation of the internal veins and channels, so the corresponding acupuncture points can be selected for cupping treatment according to the actual situation, thus playing a role in unblocking the meridians, harmonizing Qi and blood, and promoting blood circulation, so that the maternal breast distension and pain can be effectively relieved. The effectiveness of TCM treatment is varied, operable, and ideal, and it significantly improves postpartum lactation disorders and breast pain, which is highly accepted by mothers, as confirmed in most studies [4, 5].

Evidence-based medicine is a scientific way of thinking that values evidence and emphasizes clinical experience and knowledge as a referential basis for care and the best scientific evidence as a guide for care to implement a working model of targeted clinical practice and medical decision-making [6]. This model of care emphasizes that all professional decisions in clinical practice cannot simply be decided by personal experience but should be implemented based on scientific evidence. Compared with traditional medicine, evidence-based medicine has the advantages of professionalism, reliability, relevance, and practicality. Traditional nursing measures are mostly empirical nursing, mainly based on nurses' personal professional ability and working experience, lacking referenceable scientific literature, and nursing behavior lacks standardization, professionalism, and relevance, and clinical nursing effect and satisfaction need to be improved. Evidence-based TCM care is a nursing concept influenced by evidence-based medicine, and its core idea is to use scientific basis to achieve the best clinical care by adopting a series of evidence-based nursing and treatment measures in response to clinical influencing factors and nursing difficulties.

## 2. Data and Methods

### 2.1. General Information

100 parturients with postpartum breast pain treated at Taizhou First People's Hospital from January 2020 to December 2021 were selected. Among them, 51 cases received routine nursing intervention (general group, GG), and 49 cases received TCM characteristic nursing based on evidence-based medicine (comprehensive group, CG). Inclusion criteria were as follows: (1) parturient who had singleton full-term pregnancy; (2) maternal and infant immune function is good, and there is no infectious disease; (3) those who signed the informed consent form. Exclusion criteria were as follows: (1) puerpera with pregnancy complications and high-risk pregnancy; (2) deformed breast development or breast disease; (3) puerpera with significant organ dysfunction; (4) puerpera with a history of mental illness or communication disorders. The study has been approved by the Ethics Committee.

The maternal age range in the GG was 22∼35 years, with a mean age of (28.45 ± 5.47) years. The age range of the CG was 21∼35 years, with a mean age of (27.53 ± 4.95) years. There was no statistically significant difference between the two groups in terms of age, number of deliveries, and education level (*P* < 0.05), which was comparable, as shown in Table 1.

### 2.2. Nursing Methods

#### 2.2.1. In the GG

Routine nursing is mainly reflected in the following aspects: First, the patient is required to have full rest in the designated bed. Second, related matters needing attention are explained to patients with postpartum breast pain in the process of postpartum care. Third, the vital signs of patients with postpartum breast distension pain should be monitored carefully. Fourth, a series of traditional intervention measures, such as dietary intervention, should be carried out carefully according to medical advice for patients' clinical infusion and patients' selection of corresponding drugs. Finally, all patients with breast pain need to carry out ward patrol work at a fixed time, and the patient care records need to be carefully carried out every day.

#### 2.2.2. In the CG

1. An evidence-based nursing team was established to identify evidence-based issues such as psychological interventions, pain care, and complication prevention based on clinical practice experience and group discussions.
2. Medical literature databases such as Wanfang and CNKI are searched to retrieve keywords such as postpartum breast pain care and postpartum lactation volume, the existing research results retrieved are referred, and targeted TCM nursing interventions are developed according to each patient's actual situation.
3. The specific interventions are as follows: (1) *Cold Compress.* For women with swollen breasts within 1 day to 3 days, we use cold compresses on the breasts. When the room temperature is below 18∼20°C, we use a medical hand set with tap water on the breast. When the room temperature is above 18–20°C, we use the glove with tap water, put it in the refrigerator for 0.5 h, and then put it on the breast. Medical gloves are soft and can avoid the discomfort caused by cold water directly touching the skin of the mother. (2) *Acupressure*. Acupressure was performed 2 h after delivery by applying a hot towel to the mother's breasts at 43°C for 5 min and then applying Vaseline evenly to the mother's breasts. After the acupuncture points of Tan Zhong, Shao Ze, Breast Root, Shoulder Well, and Breast Middle were selected, each acupuncture point was pressed for 1 min by point massage method. In the case of postpartum stuffiness and fullness of the chest and ribs, the mother should be instructed to stay in the supine position; then, we massage around her breasts and rub her ribs lightly and select the acupoints of Taichong, Yanglingquan, Zhimen, Zhangmen, and Sanyinjiao for point massage for 1 min each; then, we select the acupoints of Spleen Yu, Liver Yu, and Diaphragm Yu on her back for Zen push massage for 2 min each. (3) *Cupping Therapy*. Cupping therapy mainly selected the puerpera Jianjing, Ganyu, Danzhong, Taichong, and other acupuncture points for cupping treatment. The puerpera first taps the Taichong point with a skin needle, and when the Taichong point shows slight bleeding or local skin reddening, then proceed to other acupuncture points for cupping treatment. During extubation, the cupping time at each point was 10 min, and cupping was performed once a day.

In the process of treating and caring for the mother, it is also necessary to communicate closely with her, to grasp the changes in her psychological state and to give her effective psychological care. The main purpose is to explain the causes of postpartum breast swelling and pain, introduce the techniques of postpartum breast care, wash the breasts with warm water, forbid the use of soap or alcohol to touch the nipples, and wear a cotton bra of appropriate size and good ventilation during breastfeeding to prevent pressure on the milk ducts that may affect lactation.

### 2.3. Observation Target

1. Numeric Rating Scale (NRS) [7] was used to evaluate maternal breast tenderness before intervention and 3 days after intervention, with a score of 0–10, 0 being no pain and 10 being severe pain. The higher the score, the more severe the maternal pain.
2. The effect of lactation in both groups was evaluated in terms of serum prolactin and total lactation after 3 days of intervention. 2 ml of fasting venous blood was collected, and it was centrifuged at 3000 r/min for 5 min; prolactin was measured using a Myriad CL-1000i fully automated chemiluminescence analyzer manufactured by Shenzhen Myriad Biomedical Electronics Co.
3. The Breastfeeding Self-Efficacy Scale-Short Form (BSES-SF) [8] was used to assess maternal breastfeeding self-efficacy before intervention and 3 days after the intervention. There are 14 items in the table, and each item is scored by Likert 1 to 5, ranging from not confident at all to always confident, with a total score of 14 to 70. The higher the score, the higher the level of self-efficacy of breastfeeding.
4. Self-rating Anxiety Scale (SAS) [9] was used to assess the subjective feelings of parturients, as a basis for measuring the severity of anxiety and its changes in treatment. There were 20 items in the scale, and a 4-level scoring method was used to evaluate the frequency of symptoms. The total score was 20–80, and the higher the total score, the higher the anxiety level. The Self-Rating Depression Scale (SDS) [10] was used to quantify the severity of maternal depressive states and changes in treatment. The scale consists of 20 items and uses a 4-point scale in which the scores of each of the 20 items are added together to obtain a total score, with the total score ranging from 20 to 80, and the higher the total score, the more severe the depression.
5. We made a nursing satisfaction questionnaire, which included scoring the quality of nursing service and the attitude of nursing staff, with a full score of 100 points. According to the score from high to low, it was divided into three grades: very satisfied (≥90 points), satisfied (60–89 points), and dissatisfied (<60 points). Nursing satisfaction rate = (very satisfied + satisfied)/total number of cases × 100%.
6. The two groups were followed up to record the situation of exclusive breastfeeding before discharge.

### 2.4. Statistical Analysis

All data were statistically analyzed using SPSS 23.0. The continuous variables such as age, NRS score, and BSES-SF score conformed to a normal distribution with their means ± SD, and *t* tests were used. The *χ*^2^ test was used to describe the number of cases and percentages of categorical variables such as number of births, literacy level, and nursing satisfaction. All statistical tests were conducted using a two-sided test, and *P* < 0.05 was considered statistically significant.

## 3. Results

### 3.1. NRS Score of Breast Swelling Pain

Three days after intervention, the NRS score of the CG was significantly lower than that of the GG (3.67 ± 0.75 vs. 5.08 ± 1.04) (*P* < 0.05), as shown in Table 2 and Figure 1.

### 3.2. Lactation Effect

3 days after intervention, the serum prolactin level in the CG was higher than that in the GG (429.65 ± 33.52 vs. 365.47 ± 36.24) and total breast lactation yield of CG was higher than of GG (435.67 ± 28.38 vs. 385.35 ± 30.41) (*P* < 0.05), as shown in Table 3.

### 3.3. BSES-SF Score of Breastfeeding Self-Efficacy

Three days after intervention, the BSES-SF score of maternal breastfeeding self-efficacy was higher in both the groups and the BSES-SF score of maternal breastfeeding self-efficacy in the CG was significantly higher than that in the GG (59.00 ± 6.70 vs. 50.65 ± 8.37) (*P* < 0.05), as shown in Table 4.

### 3.4. SAS Score and SDS Score

Three days after intervention, the SAS score and SDS score in the CG were significantly lower than those in the GG (*P* < 0.05), as shown in Table 5.

### 3.5. Nursing Satisfaction

The nursing satisfaction of women in GGG was 74.51% (40/51), and that of women in CG was 91.84% (45/49), which was significantly higher than that of GG (*P* < 0.05), As shown in Table 6.

### 3.6. Exclusive Breastfeeding Rates

The rate of exclusive breastfeeding in the CG was 85.71%, which was higher than that in the GG (62.75%), and the difference was statistically significant (*χ*^2^ = 8.672, *P*=0.003).

## 4. Discussion

Breast milk is the best food for babies, and breastfeeding has many benefits for both babies and mothers. For mothers, breastfeeding reduces weight retention, which means it can help control weight, and, in addition, breastfeeding can reduce the risk of breast cancer and diabetes and it also allows mothers to deeply feel the happy feelings of motherhood and promotes mutual emotional communication between the mother and the baby [11, 12]. For infants, breast milk is nutritionally comprehensive and in some ways more advantageous than formula. And, it can also establish a healthy intestinal microecology in babies, reducing the risk of allergies and various inflammatory conditions [13, 14]. Overall, breastfeeding is safer, is more convenient, and can increase parent-child bonding [15]. In addition, breastfeeding is one of the best investments to save babies' lives, improve individual and national health, and increase social and economic development. A study by the British Medical Journal, The Lancet, showed that if optimal breastfeeding were practiced globally, more than 823,000 children and 20,000 mothers could be prevented from dying each year and economic losses could be reduced by approximately $302 billion per year. This shows that supporting breastfeeding is undoubtedly the right move for individuals, families, and society as a whole [16, 17]. Despite the increasing awareness of breastfeeding, there are still some new mothers who have no choice but to give up due to breast swelling and pain. In the early stage of breastfeeding, hormones such as prolactin and adrenocorticotropic hormone of the maternal organism are important for lactation regulation and the incidence of postpartum breast swelling and pain is higher. Postpartum breast distension is a common phenomenon among new mothers, and breast distension, nipple pain, and milk stagnation not only affect the postpartum recovery of the mother but also have a negative impact on the newborn's breastfeeding [18, 19].

Evidence-based care is a service based on evidence-based medicine that follows up on the professional competence and work experience of nursing staff to provide targeted care for patients' needs. It includes three elements: (1) the most appropriate nursing research base available; (2) the personal skills and clinical experience of the nursing staff; (3) the actual situation, sense of values, and wishes of the patient [20]. In addition, TCM has always attached importance to nursing care and based on the physiology and pathology of TCM organs and meridians, Qi, blood, and fluids, a set of discriminative nursing methods from theory to clinical practice and operational techniques with TCM characteristics, such as cupping therapy, fumigation therapy, compressing method, and Chinese herbal medicine method, massage, have achieved good efficacy in several fields [21, 22]. Arora et al. [23] concluded that painful breast swelling due to sudden increase in milk volume, lymphatic and vascular engorgement, and interstitial edema caused by inadequate breastfeeding and (or) milk duct obstruction can be treated with cold cabbage leaves and alternating hot and cold compresses, but cold compresses are more effective than cold cabbage leaves in relieving breast swelling and pain. Cupping therapy works by simply stimulating the skin with suction to increase local circulation of blood and lymph and relieve painful muscle tension [24]. Yazdanpanahi et al. [25]showed that both cupping therapy and acupressure were effective in reducing postpartum low back pain in primiparous women, but the pain intensity was significantly reduced in the cupping therapy group. The results of this study also showed that the NRS score of the CG (3.67 ± 0.75) was significantly lower than that of the GG (5.08 ± 1.04), suggesting that mothers receiving TCM specialty care were more effective in relieving postpartum breast tenderness compared to conventional care, similar to Arora et al. [23] and Yazdanpanahi et al. [25] studies.

Cold compresses reduced venous filling and interstitial engorgement in the breast, and the mothers felt less self-induced distension and pain and were comfortable and receptive to cold compress care compared with the traditional hot compress method used in the past within 1 to 3 d. This result suggests that TCM care can also promote milk discharge, increase maternal lactation after delivery, and improve the rate of exclusive breastfeeding. Chen et al. [26] showed that acupressure combined with breast massage significantly shortened the onset of lactation, increased lactation volume, effectively improved breast distension, and increased breastfeeding rate. The present study is consistent with the study of Chen et al. [26]. Breast massage is a common tool in postpartum care, which mainly promotes blood and lymphatic circulation inside the breast, unblocks the milk ducts, and then drains the milk accumulated in the ducts, to reduce the risk of maternal breast distension and pain. Clinical massage is mainly used to massage maternal breasts with professional massage techniques, which stimulate the peripheral nerves of the breast and induce the pituitary gland to release large amounts of prolactin, thus shortening the duration of colostrum secretion and increasing the amount of lactation [4, 27]. At the same time, breast massage stimulates maternal breasts and nipples with the help of kneading and lifting, which can improve the blood circulation of breasts and make them soft, and the nipples and nipple necks can be freely bent to facilitate newborns to take them, guarantee the sucking effect and facilitate the emptying of milk, and promote exclusive breastfeeding.

## 5. Strengths and Limitations

In the context of the continuous reform and innovation of the medical model, the functions of nursing staff have also changed, from being traditional implementers of medical device orders to comprehensive caregivers of patients in the postoperative period. Evidence-based nursing requires people to follow scientific principles and basis in medical practice, adopt targeted TCM evidence-based nursing methods, instruct mothers on the correct concept of breastfeeding, and focus on psychological interventions, health education, and pain relief which have important clinical consequences in improving maternal breastfeeding rate. The nursing staff paid enough attention to the various opinions of the mothers and used various methods in a timely manner to solve the various problems that existed between them, which made the satisfaction of the mothers with the nursing care increase. There is still room for improvement in this study, such as expanding the scope of the study and increasing the sample size by combining multiple medical institutions.

## 6. Conclusions

With the improvement of modern medicine, it has become the mainstream awareness in many countries to promote breastfeeding; after all, it has been proven that children who have been breastfed have better physical resistance and other abilities. However, the incidence of postpartum breast pain and lactation is high and requires effective nursing intervention. One study [28] evaluated the effectiveness of interventions such as glycerin gel dressings, nonpharmacologic topical treatments (e.g., lanolin), breast milk compression, and multipurpose nipple ointment in relieving or reducing nipple pain and found that for most women, regardless of the treatment used, nipple pain was reduced to a mild level after approximately 7 to 10 days postpartum. The women in this study who were given evidence-based TCM care experienced significant reduction in breast tenderness and lactation after 3 days of treatment. Evidence-based TCM care can significantly reduce postpartum breast tenderness, increase milk production, improve exclusive breastfeeding, and help relieve emotional distress.

## Figures and Tables

**Figure 1:** Comparison of NRS scores of breast swelling pain between the two groups.

**Table 1:** General information.

Information	GG	CG	*t*/*χ*^2^ value	*P* value
Age (years)				
Range	22∼35	21∼35		
Mean ± SD	28.92 ± 3.69	28.22 ± 3.69	−0.945	0.347
Production time			0.360	0.548
Pluripara	27	23		
Unipara	24	26		
Cultural level			0.027	0.986
Primary and below	11	10		
Junior/senior high school	26	25		
Bachelor degree or above	14	14		
Delivery way			0.818	0.366
Natural birth	32	25		
Cesarean delivery	19	24		
Gestational age (weeks)			0.820	0.415
	38∼42	38∼42		
	39.61 ± 1.17	39.81 ± 1.27		

**Table 2:** NRS score of breast swelling pain (points ± SD).

Group	*N*	Before intervention	3 days after intervention
GG	51	7.86 ± 0.87	5.08 ± 1.04^*∗*^
CG	49	7.59 ± 1.29	3.67 ± 0.75^*∗*^
*t* value		−1.235	−7.751
*P* value		0.220	<0.001

*Note*. ^*∗*^Comparison of 3 days after intervention with before intervention, *P* < 0.05.

**Table 3:** Comparison of lactation effects between the two groups.

Group	*n*	Serum prolactin (ng/L)	Total breast lactation yield (mL)
GG	51	365.47 ± 36.24	385.35 ± 30.41^*∗*^
CG	49	429.65 ± 33.52	435.67 ± 28.38^*∗*^
*t* value		9.184	8.547
*P* value		<0.001	<0.001

*Note*. ^*∗*^Compared with before intervention, *P* < 0.05.

**Table 4:** BSES-SF score of breastfeeding self-efficacy (points ± SD).

Group	*n*	Before intervention	3 day after intervention
GG	51	38.65 ± 5.41	50.65 ± 8.37^*∗*^
CG	49	36.90 ± 6.12	59.00 ± 6.70^*∗*^
*t* value		−1.515	5.497
*P* value		0.133	<0.001

*Note*. ^*∗*^Compared with before intervention, *P* < 0.05.

**Table 5:** SAS score and SDS score (points ± SD).

Group	*n*	SAS score		SDS score	
		Before intervention	3 day after intervention	Before intervention	3 day after intervention
GG	51	57.29 ± 7.31	41.10 ± 9.46^*∗*^	56.25 ± 9.70	40.88 ± 8.71^*∗*^
CG	49	59.18 ± 8.45	36.45 ± 7.99^*∗*^	56.20 ± 10.42	36.80 ± 7.75^*∗*^
*t* value		1.166	−2.65	−0.025	−2.475
*P* value		0.246	0.009	0.980	0.015

*Note*. ^*∗*^Compared with before intervention, *P* < 0.05.

**Table 6:** Nursing satisfaction.

Group	*n*	Very satisfied	Satisfied	Dissatisfied	Rate
GG	51	19	19	13	74.51%
CG	49	27	18	4	91.84%
*χ * ^2^ value					6.146
*P* value					0.046

## Data Availability

The data used to support the findings of this study are available from the corresponding author upon request.
